This article has been retracted.

# Image Observation Study on Improving the Effectiveness of Muscle Strength Training for Sprinters

**DOI:** 10.1155/2022/4987782

**Published:** 2022-07-25

**Authors:** Yimin Zou, Liming Han

**Affiliations:** ^1^Ministry of Culture, Sports and Labour, Gannan Healthcare Vocational College, Ganzhou, Jiangxi 341000, China; ^2^College of Physical Education, Xingtai University, Xingtai, Hebei 054001, China

## Abstract

In order to solve the problem of improving the effectiveness of muscle strength training for sprinters, this paper presents a study using image observation technology. The main content of this technology research is to determine the experimental object and method according to the image observation and muscle characteristics. Through the data processing and other processes, it is concluded that the image observation technology has a high accuracy in the observation of muscle movement patterns. The experimental results show that when the relationship number *r* = 0.99, the average error of prediction is 0.09, and the image observation technology has a high accuracy in the observation of muscle movement. *Conclusion*. It is proved that the technical research of image observation is effective and accurate for improving the training of sports muscle strength of sprinters.

## 1. Introduction

In the process of the steady development of China's sports cause, the emphasis on training has gradually increased, as has the sprint team. When carrying out the special strength training of the sprint team (Figure 1), it is necessary to adjust the traditional training methods, so that the special strength of the sprint can play a role together with the general strength training, improve the performance of the sprinters, and hope to have some help for the development of China's sports school athletes [1]. For a long time, traditional strength training has played a key role in enhancing the strength of athletes' upper and lower limbs, and the sprint performance has been continuously improved, but our elite athletes have hardly achieved good results in sprint events [2]. In recent years, scholars have strengthened the theoretical research of strength training, especially carried out a series of experiments on the shortcomings of traditional strength training, and formed a corresponding comparison between the new strength training methods and traditional strength training. Strength training refers to the ability of human neuromuscular system to overcome or resist resistance during work.

Traditional strength training has been playing an important role in improving sprint performance. It is mainly based on the principle of excess recovery to do incremental resistance strength training to improve muscle strength. In the process of exercise, the ability of human neuromuscular system to overcome and resist resistance at work is simply based on increasing load to enhance strength. Traditional strength training pays attention to the development of a single muscle. When muscle strength is enhanced, muscle volume is also increasing. Its basic methods mainly include dynamic isometric contraction training, static isometric contraction training, isometric contraction training, super isometric contraction training, and circular training, which are widely used in sprint strength training [3].

Scientifically and reasonably designing strength training, developing the strength ratio of the flexor and extensor muscles in the medulla, the coordinated and balanced development of the strength of the upper and lower limbs, and the contraction ability of the muscles of the metacarpophalangeal and ankle joints are the most important to improve the performance of sprint. In the traditional strength training, the general strength training and special strength training are applied repeatedly, which enhances the muscle strength of athletes and lays a certain foundation for the improvement of performance. We should pay more attention to the strength training of the extensor group instead of the flexor group and from the training of maximum strength to the training of fast strength and strength endurance. This training guiding ideology is more in line with the characteristics of modern sprint sports and provides more pertinence and scientificity for better improving sprint performance [4].

## 2. Literature Review

With the country's vigorous sports undertakings, under the current background, strength training has an important impact on the improvement of sprint performance; the world record of 100 m performance especially has been broken repeatedly. We should strengthen strength training and combine it with sprint technology. In strength training, it is necessary to design strength training methods and means suitable for project characteristics and sports biomechanics characteristics according to the working forms and force characteristics of sprint technical movements. Traditional strength training has always played an important role in improving sprint performance, but there are also some shortcomings in traditional strength training. We should make up for them. It is the all-round development of Chinese athletes' muscle strength to improve their sprint performance. Strength training can effectively enhance the contractility of muscles, improve the resistance of human neuromuscles to external activities, and effectively exercise the human skeletal system [5]. High school physical education teachers should constantly guide students to carry out strength training, ensure the explosive power of muscle groups through the training of outburst, reaction, and starting strength, emphasize the integrity and continuity, and establish a perfect evaluation and monitoring system to timely point out the lack of training of students and improve the sprint training effect, so as to enable students to develop a good physique and promote physical health. The development level of athletes' muscle strength quality and the good coaxiality and coordination among active muscle, antagonistic muscle, and synergetic muscle in sports are one of the main factors to measure sprint technology and determine sports performance. The ultimate purpose of selecting strength training methods is to effectively develop the strength of the muscles and muscle groups participating in special sports, make them work in line with the characteristics of special technology, and form a strength quality system with special projects as the core, so as to enhance the special ability of athletes and further improve their special performance. Strength training is the source of all kinds of sports. Sprint is a periodic speed strength event. Muscle strength and speed are directly related to running speed. Double the running speed and quadruple the resistance; that is to say, the faster the speed is, the greater the muscle strength is required. Therefore, if you want to improve the speed, you must enhance the muscle strength, so strength is very important to improve the sprint performance.

In view of the above problems, this paper proposes an image observation study to improve the effectiveness of muscle strength training for sprint athletes [6]. The main content of this study is to determine the experimental objects and methods based on image observation and muscle characteristics, and through data processing, it is concluded that the image observation technology has a high accuracy in the observation of muscle movement patterns. Accurate observation of the impact of strength training on the athletes' muscles helps in formulating a targeted way of strength training for athletes and providing a scientific basis for improving sprint performance.

## 3. Research Methods

### 3.1. Image Observation and Muscle Characteristics

Muscle (especially skeletal muscle) contraction is the driving force for human body to generate movement. In order to understand human movement and reveal the mechanical law of movement, it is necessary to study the structure, function, and characteristics of human muscle [7]. Due to the complexity and diversity of the movement process, the study of muscle function and characteristics in the movement process is a complex and arduous task, especially how to simultaneously obtain a variety of information from a single muscle in the human body and carry out multilevel comprehensive processing is still a difficult problem to be solved.

Surface electromyographic signal (SEMG, hereinafter referred to as SEMG) is an electrophysiological signal obtained from the skin surface. It is a common method to study the activities of the neuromuscular system and is widely used in biomechanics, rehabilitation medicine, and other fields [8]. EMG signal is the superposition of action potentials generated by many motor units in muscle fibers during contraction. Its time-frequency characteristics can quantitatively reflect the characteristics and laws of muscle function, muscle strength level, multimuscle group coordination, etc. However, EMG signal is vulnerable to various potential factors, such as electrode position, muscle type, and adjacent muscle interference, which restrict the application of EMG signal in muscle evaluation.

Different from EMG signals, muscle tone signals (MMG, also translated into muscle motion signals) are signals generated by the lateral vibration of muscle fibers during muscle contraction and also contain the functional state information of muscles [9]. EMG reflects the electrical activity of the moving unit, while MMG reflects the mechanical activity of the moving unit. MMG can be collected by a variety of sensors, including piezoelectric sensors, micro microphones, and acceleration sensors. Many studies have compared EMG with MMG, and the results show that MMG has different time-frequency characteristics from EMG. MMG combined with EMG can provide complementary information about muscle movement.

Muscle contraction will cause changes in muscle morphology, so changes in muscle morphology can directly reflect the state of muscle activity. Various clinical imaging methods, including CT, MRI, and ultrasound, have been used to study muscle morphological changes. Among them, ultrasonic imaging (US) has the characteristics of nondestructive, real time, and easy to use, which has been more applied [10]. Since the 1990s, researchers have tried to use morphological parameters extracted from ultrasound images to reflect the changes of muscle function. These parameters include muscle thickness, cross-sectional area, muscle fiber length, and feather angle, which are closely related to muscle function. Due to the real-time nature of US, it can be applied to various forms of muscle movement, including isometric movement, standing, walking, and muscle contraction caused by electrical stimulation [11]. All these studies show that US, that is, simple, nondestructive, and real time, can measure muscle contraction, which is difficult to achieve by other existing technologies. Compared with EMG, US has the advantage that it is not affected by adjacent muscles and can measure deep muscles. In some cases, it is more sensitive to changes in muscle contraction. Among the muscle morphological parameters, cross-sectional area (CSA) is of special significance, which determines the strength of muscle. However, most studies focus on the influence of age, training, and other factors on CSA. Few studies have studied the changes of CSA during muscle dynamic contraction. The main reason is that it is a difficult problem to automatically obtain CSA from continuous ultrasound images.

EMG, MMG, and US, respectively, reflect the electrical, mechanical, and morphological changes of muscle movement and can provide complementary information for the study of muscle movement. Previous studies mostly combined EMG with ultrasonic MMG. But so far, few studies have combined the three to further reveal the internal physiological mechanism of muscle continuous movement. Based on the above considerations, the author developed a multichannel motion signal acquisition system, which can synchronously collect US, EMG, MMG, joint angle, and torque signals. In addition, in order to track the continuous change of CSA, the author also developed a new image tracking algorithm to achieve the automatic acquisition of CSA. Using this system, this study studied the isometric contraction of rectus femoris (RF) during knee extension, analyzed the characteristics of various signals collected, and preliminarily established a new method for multimodal study of muscle motion characteristics [12].

### 3.2. Experimental Process

#### 3.2.1. Test Object and Method

A total of 9 subjects participated in the experiment, including 6 males and 3 females. During the experiment, the subjects sit on the experimental chair of the isokinetic muscle strength test system and fix the body with safety belts. The hip and knee joints are kept at 90°, and the lower leg is fixed on the rotating shaft through the fixing belt, so the isometric contraction movement of knee joint extension can be carried out [13].

Before the beginning of the experiment, a rectus femoris image was collected as a reference when the subjects were relaxed. Then, the subjects completed two isometric knee extension movements lasting for 6 s to determine the maximum arbitrary contraction (MVC) of the muscle and defined MVC as the maximum amplitude of isometric contraction of the muscle [14]. Then, the subjects did several warm-up exercises to familiarize themselves with the experimental rules. After 5 min of rest, the subjects will complete isometric muscle contraction under continuous increasing load, and the torque requirements will increase linearly from 0%MVC to 90%MVC for 6 s. In the experiment, the knee joint extension torque generated by the subjects will be detected by the system, and its time-varying waveform will be displayed on the display screen in front of the subjects in real time. The standard torque waveform (from 0%MVC to 90%MVC within 6 s) will also be displayed at the same time. The subjects will adjust their actions to make the torque waveform generated by themselves match the standard waveform as much as possible. The subjects will repeat the experiment for 3 times and rest for 5 min between every two adjacent experiments [15].

During the experiment, ultrasound images of rectus femoris muscle were obtained by ultrasound scanner. The ultrasonic probe is fixed above the thigh through a self-made multiangle bracket, and its long axis is perpendicular to the direction of the thigh. The video output of the ultrasonic equipment is captured by the video acquisition card, and the sampling frequency is 25 frames/s. Two surface EMG electrodes are attached to the rectus femoris muscle abdomen, along the muscle fiber direction, at the positions on both sides of the probe, and the reference electrode is attached to the knee. The acceleration sensor is pasted on the muscle surface near the ultrasonic probe with double-sided tape to collect MMG signals. EMG and MMG are amplified by a self-made amplifier with a gain of 2000, and then, bandpass filtering of 10~400 Hz and 5~100 Hz is performed, respectively, and finally digitized by a data acquisition card with a sampling frequency of 1 kHz. The torque signal output by the isokinetic muscle strength tester is also sampled by the data acquisition card, and the display, synchronous acquisition, and storage of all signals are completed by the self-developed software, and the saved data will be further analyzed and processed [16].

#### 3.2.2. Data Processing

EMG and MMG signals of each subject were processed offline by software. The EMG and MMG are divided into 256 MS segments according to time, and the time center of each segment is aligned with the corresponding ultrasonic image acquisition time [17]. Since the sampling frequency of the image is 25 frames/s, there is a certain coincidence between the two adjacent segments of EMG and MMG. Then, the root mean square value of each segment is calculated as the time domain characteristic index of EMG and MMG. By definition, RMS is calculated as follows.

(1) $$\begin{array}{c} \text{RMS}=\sqrt{\frac{1}{N}\overset{N}{\underset{i=1}{\sum }}x_{i}^{2}} \end{array}$$

In the global transformation, the transformation parameters are composed of the global scale, translation, and rotation transformations of two images, and the global affine transformation function *T* = *ψ* [*x*, *y*, 1] *T*, where *x* and *y* are image coordinates and *ψ* is an affine transformation matrix of 3 × 3. If *a* and *B* are the images to be matched, the global mutual information is calculated as follows.

(2) $$\begin{array}{c} \text{MI}=I\left(A;T\left(B\right)\right)=H\left(p_{A}\left(i_{A}\right)\right)+H\left(p_{T\left(B\right)}\left(i_{B}\right)\right)-H\left(p_{A,T\left(B\right)}\left(i_{A},i_{B}\right)\right)=\iint_{I\left(A\right),I\left(B\right)}\;p_{A,T\left(B\right)}\left(i_{A},i_{B}\right)\mathrm{lg}\left(\frac{p_{A,T\left(B\right)}\left(i_{A},i_{B}\right)}{p_{A}\left(i_{A}\right)p_{T\left(B\right)}\left(i_{B}\right)}\right)\text{d}i_{A}i_{B}. \end{array}$$

Continue to perform local transformation on the results after global transformation, and use 2D spline function TL (B′) to describe the local transformation [18]. *M* and *N* are the number of horizontal and vertical control points, respectively. In the third-order neighborhood of the control point, the transformation function can perform third-order spline interpolation based on the transformation result of the control point, and formula (3) is calculated.

(3) $$\begin{array}{c} P\left(i,j\right)=\overset{3}{\underset{\mu =0}{\sum }}\overset{3}{\underset{\gamma =0}{\sum }}\beta_{\mu }\left(u\right)\beta_{\gamma }\left(v\right)P_{c}\left(m+\mu ,n+\gamma \right). \end{array}$$

Leave one test is used to test the accuracy of multiparameter linear estimation. Each time, the data of one subject is left for test, and the data of other subjects are used as the linear regression coefficient to calculate the coefficient. Then, the fitting coefficient is used to predict the torque of the left subject, and the error with the real torque is calculated. This is repeated many times, so that each subject is left alone for a test, and finally calculate the average prediction error [19].

## 4. Result Analysis

During muscle contraction, typical joint torque signals are shown in Figure 2. The circle in the figure represents the joint torque generated by the subject, and the solid line represents the standard torque signal used to guide the subject [20]. These two signals will be displayed in front of the subject in real time in the experiment.

The original waveform and RMS amplitude of EMG and MMG are shown in Figures 3 and 4. In order to study the relationship between RMSEMG, RMSMMG, and joint torque, curves are drawn in the same coordinates, as shown in Figure 5 [21].

100 ultrasound images were processed manually and by image algorithm. The results of ICC analysis were 0.987 (*P* < 0.0001). The results show that the image algorithm can accurately track the muscle boundary and basically achieve the same effect as manual processing. The relationship between the overall average value of different parameters and joint torque is composed of the upper and lower limits of the data average standard error se, and the solid line is a cubic polynomial fitting curve [22]. Image tracking algorithm can automatically extract the boundaries of rectus femoris muscle in all images and calculate the corresponding CSA. The relationship between CSA and joint torque in this experiment changes. The cubic polynomial curve is used for fitting, and the fitting results are also displayed.

EMG is a traditional method to study muscle activity. A large number of researchers have deeply discussed the relationship between EMG and muscle strength. At present, it is generally believed that the relationship between the two is nonlinear and affected by many factors. It is difficult to accurately estimate the muscle force only from the EMG of a single channel. MMG is a signal produced by the lateral vibration of muscle fibers during muscle contraction, which is different from EMG in nature.

Combining the three parameters of RMSEMG, RMSMMG, and CSA, carry out multiparameter linear fitting for the joint torque. The fitting results are compared with the actual measurement. The abscissa is the actual measured torque, the ordinate is the fitted torque, the circle is the fitting data point, and the solid line is the reference line with a slope of 1. The correlation coefficient *R* = 0.99 is obtained, and the average error of prediction is 0.09 through the leave one test, as shown in Table 1.

## 5. Conclusion

In order to solve the problem of improving the effectiveness of muscle strength training for sprinters, this paper presents a study using image observation technology. The main content of this technology research is to determine the experimental object and method according to the image observation and muscle characteristics. Through the data processing and other processes, it is concluded that the image observation technology has a high accuracy in the observation of muscle movement patterns. Accurately observe the impact of strength training on Athletes' muscles, so as to formulate a targeted way of strength training for athletes and form a strength quality system with special projects as the core, so as to enhance athletes' special ability and further improve their special performance, which provides a scientific basis for improving sprint performance and is very important for improving sprint performance.

## Figures and Tables

**Figure 1:** Weight training.

**Figure 2:** Waveform of joint torque with time during muscle contraction.

**Figure 3:** EMG waveform.

**Figure 4:** MMG waveform.

**Figure 5:** Relationship between EMG root mean square amplitude and joint torque.

**Table 1:** Fitting results.

Project	Numerical value
Slope	1
Correlation coefficient	0.99
Forecast average error	0.09

## Data Availability

The data used to support the findings of this study are available from the corresponding author upon request.
